RETRACTED

# Effect of Enalapril Combined with Bisoprolol on Cardiac Function and Inflammatory Indexes in Patients with Acute Myocardial Infarction

**DOI:** 10.1155/2022/6062450

**Published:** 2022-08-18

**Authors:** Kaiyue Huang, Yubin Zhang, Fulin Yang, Xue Luo, Weiying Long, Xingzhi Hou

**Affiliations:** Internal Medicine-Cardiovascular Department, The People's Hospital of Yue Chi, No. 22, Jianshe Road East, Yuechi County, Sichuan Province, China

## Abstract

**Objective:**

The use of enalapril in combination with bisoprolol in patients with acute myocardial infarction (AMI) was studied for its effect on cardiac function and inflammatory parameters.

**Methods:**

Sixty-two cases of AMI patients admitted to our clinic from November 2019 to November 2021 were selected for the study and grouped according to the random number table method, those enrolled were given conventional treatment such as oxygenation, absolute bed rest, and sedation, and administered low molecular heparin, aspirin, atorvastatin calcium tablets, clopidogrel, and nitrates. The control group (31 cases) was treated with enalapril maleate folic acid tablets, and the treatment group (31 cases) was treated with bisoprolol fumarate tablets on top of the control group, and the efficacy, adverse effects, cardiac function, inflammatory indexes, and oxidative stress indexes of the two arms were contrasted.

**Results:**

The incidence of adverse reactions in the therapy cohort was 12.90% higher than that in the controlled arm, but the discrepancy was not medically relevant (*P* < 0.05). The SOD level was larger than the concentration in the corresponding drug therapy group, and the MDA level was lower than the concentration in the respective test cases (*P* < 0.05); the incidence of 12.90% adverse reactions in the treatment period was lower than that of 16.13% in the specific drug therapy group, but the variance was not scientifically evident (*P* > 0.05).

**Conclusion:**

Enalapril application combined with bisoprolol in AMI patients is beneficial to boost the efficacy, promote the improvement of cardiac function, reduce the inflammatory response, and improve the oxidative stress with fewer adverse effects, which can ensure the therapeutic security.

## 1. Introduction

Acute myocardial infarction (AMI) is one of the common and frequently-occurring diseases in the clinic. Patients often present with severe and persistent pain behind the sternum, accompanied by symptoms such as heart failure, arrhythmia, and circulatory function decline [1]. Myocardial infarction is one of the most common clinical causes of chronic heart failure, and more than 50% of heart failure patients die within 5 years of diagnosis. Studies have found that once AMI occurs, a series of changes can occur in the structure and morphology of the left ventricular infarcted area and the noninfarcted area, which is called left ventricular remodeling [2]. One of the common complications of AMI is cardiac insufficiency, which can increase the mortality rate of patients. Therefore, the prevention of cardiac insufficiency should be the main content in the clinical treatment of AMI. The first step in the treatment of AMI is to quickly identify the disease through biological indicators, electrocardiogram, etc., and give drugs to relieve ischemic pain, evaluate hemodynamic indicators, and correct possible abnormalities. Although it has been reported that the use of drug therapy during hospitalization can prolong the survival time of AMI patients and help reduce the mortality rate, problems such as recurrence, cardiac structural reconstruction and cardiac function changes still exist [3]. Angiotensinase inhibitor (ACEI) can inhibit the progressive left ventricular remodeling of AMI. As an ACEI, enalapril can control the scope of myocardial infarction to achieve the purpose of reducing mortality [4, 5]. *β*-blockers are beneficial to reduce the recurrence of myocardial ischemia, and bisoprolol, as a *β*-blocker, can effectively reduce the risk of arrhythmia. The efficacy of the combination of the two drugs in the treatment of AMI has been clinically recognized, but there are few reports on the effect of the combination therapy on the inflammatory indexes in patients with AMI. This time, 62 AMI patients admitted to our hospital from November 2019 to November 2021 were selected to study the effects of enalapril combined with bisoprolol on cardiac function and inflammatory indexes in AMI patients. The report is as follows.

RETRACTED

## 2. Materials and Methods

### 2.1. General Materials

Sixty-two patients with AMI admitted to our hospital from November 2019 to November 2021 were selected for the study, and the inclusion criteria were (1) all met the diagnostic criteria for AMI in the Expert Consensus on Integrated Chinese and Western Medicine Treatment of Acute Myocardial Infarction [6]; (2) age >18 years; (3) New York Heart Association (NYHA) class II–IV; (4) onset to admission time <6 h; (5) patient informed consent; (6) complete patient medical records and other information. Exclusion criteria: (1) combination of malignancy; (2) combination of hepatic and renal insufficiency; (3) combination of psychiatric or hematologic disorders; (4) combination of severe atrioventricular block; (5) allergy to this study drug; (6) presence of shock symptoms. The control group (31 cases) consisted of 18 males and 13 females, aged 48–81 years, with a mean of (60.97 ± 2.48) years; infarct sites: 13 cases in the inferior wall, 7 cases in the anterior interstitial wall, 8 cases in the anterior wall, and 3 cases in the extensive anterior wall, according to the random number table method. In the treatment group (31 cases), there were 16 males and 15 females, aged 51–78 years, with a mean of (60.86 ± 2.52) years; infarct sites: 14 cases in the inferior wall, 8 cases in the anterior interstitial wall, 7 cases in the anterior wall, and 2 cases in the extensive anterior wall. No noticeable discrepancy was detected when comparing the data of the two types of groups, *P* > 0.05. This study was approved by the ethics committee.

### 2.2. Methods

All the participants were given routine treatment such as oxygen inhalation, absolute bed rest and sedation, low molecular weight heparin (Shenzhen Saibaoer Bio-Pharmaceutical Co. Ltd.; National Medicine Zhunzi H20060191), aspirin (Heilongjiang Fuhe Pharmaceutical Group Co. Ltd.; Sinopharm approved H23023494), atorvastatin calcium tablets (Guangdong Dongguang Pharmaceutical Co. Ltd.; Sinopharm H20213513), clopidogrel (Shandong New Times Pharmaceutical Co. Ltd.; Sinopharm H20173366), and nitrates treat. On this basis, the control group was additionally treated with enalapril maleate and folic acid tablets (Shenzhen Osa Pharmaceutical Co., Ltd.; National Medicine Zhunzi H20103724; enalapril maleate 10 mg, folic acid 0.4 mg) at a dose of 5 mg/time–10 mg/time, 2 times a day. The treatment group was additionally treated with bisoprolol fumarate tablets (Beijing Huasu Pharmaceutical Co. Ltd.; Guoyao Zhunzi H20023132; 2.5 mg) on the basis of the control group, the dose ranged from 2.5 mg/time to 5.0 mg/time, 4 times a day Second-rate. All participants received treatment for 3 months.

### 2.3. Observation Indexes

#### 2.3.1. Treatment Effect

The treatment was evaluated by NYHA cardiac function grading 3 months after treatment: disappearance of arrhythmia and heart failure, reduction of NYHA cardiac function grading ≥2 or normal cardiac function test results were considered effective; significant improvement of arrhythmia and heart failure and reduction of NYHA cardiac function grading I were considered effective; not meeting the above criteria were considered ineffective. The total effective rate = the number of cases (effective + effective)/sample number × 100%.

#### 2.3.2. Cardiac Function

Echocardiography was performed 1 day before treatment and 3 months after treatment. The equipment used a UGU-100 color Doppler ultrasound system (Shenzhen Aosheng Medical Technology Co. Ltd.; Guangdong Machinery Note 20212060678) to measure left ventricular end-diastolic phase Left ventricular end-diastolic diameter (LVED), left ventricular ejection fraction (LVEF), left ventricular end-systolic diameter (left ventricular end-systolic diameter), and left ventricular mass index (LVM).

RETRACTED

#### 2.3.3. Inflammation Indicators

3 ml fasting venous blood was collected from patients 1 day before treatment and 3 months after treatment, and after centrifugation (3500 r/min, time 10 min, radius 14 cm), the supernatant was taken and stored at −20°C for inspection; equipment: EC9400 automatic biochemical analyzer (Guangzhou Exxon Biotechnology Co., Ltd.; Guangdong Machinery Standard 20152221248) and MR-96A Type Microplate Reader (Shenzhen Mindray Biomedical Electronics Co. Ltd.; Guangdong Machinery Standard 20192220393). The serum level of interleukin-6 (IL-6) was determined by enzyme-linked immunosorbent assay; the serum *N*-terminal natriuretic peptide precursor (NT-) was determined by the electrochemiluminescence double-antibody sandwich method. The proBNP level and serum C reactive protein (CRP) level were determined by turbidimetry; the kits were all provided by Shanghai Zhicheng Biotechnology Co. Ltd., and the above tests were performed in strict accordance with the kit instructions.

#### 2.3.4. Oxidative Stress

3 ml fasting venous blood was collected from patients 1 day before treatment and 3 months after treatment, and the supernatant was collected after centrifugation (speed 3000 r/min, time 10 min, radius 10 cm) for testing; EC9400 automatic biochemical analyzer (Guangzhou Exxon Biotechnology Co., Ltd.; Guangdong Machinery Note 20152221248) was used, and serum levels of superoxide dismutase (SOD) and malondialdehyde (MDA) were determined by radioimmunoassay.

#### 2.3.5. Adverse Reactions

The occurrence of hypotension, sinus bradycardia, cough, and rash in patients was recorded, and the incidence was calculated.

### 2.4. Statistical Analysis

The study data were analyzed by SPSS19.0 software, and the measurement data (conforming to normal distribution) and count data were expressed as (±*s*) and %, respectively, by *t* and *χ*^2^ tests. *P* < 0.05 means the discrepancies were of statistical importance.

## 3. Results

### 3.1. Contrast of the Therapeutic Efficiency among the Two Sets of Groups

The aggregate effective rate of 93.55% in the treatment cohort was superior to 67.74% in the control cohort (*P* < 0.05) (Figure 1).

### 3.2. Cooperation of Cardiac Functionality between the Two Arms

Compared with the levels of LVEF, LVED, LVES, and LVM, there was no significant difference between the two groups on the first day of treatment (*P* > 0.05). The level of LVM was lower (*P* < 0.05); the level of LVEF in the treatment group was higher than that in the control group 3 months after treatment, and the levels of LVED, LVES, and LVM were lower than those in the control group (*P* < 0.05), as shown in Figure 2.

RETRACTED

### 3.3. Comparison of Inflammatory Indexes between the Two Groups

Compared with the levels of NT-proBNP, CRP, and IL-6, there was no significant difference between the two groups on the first day of treatment (*P* > 0.05). The levels of IL-6 were lower (*P* < 0.05); the levels of NT-proBNP, CRP, and IL-6 in the treatment group were lower than those in the control group 3 months after treatment (*P* < 0.05), as shown in Figure 3.

### 3.4. Oxidative Stress Index Contrast between the Two Sets of Groups

Comparing the levels of SOD and MDA, there was no significant difference between the two groups on the first day of treatment (*P* > 0.05); the SOD level in the treatment group was higher than that in the control group 3 months after treatment, and the MDA level was lower than that in the control group (*P* < 0.05), as shown in Table 1.

### 3.5. Adverse Reaction Situation Contrasts by Two Groups

The occurrence rate of 12.90% adverse reactions in the therapy cohort was lower than that of 16.13% in the reaction cohort, but the discrepancy was not statistical sense (*P* > 0.05) (Table 2).

## 4. Discussion

AMI has a high incidence in China, formed by the development of chronic heart failure; patients mostly show symptoms such as shortness of breath and dyspnea, and clinical examination reveals an enlarged left ventricle with cardiogenic shock or pulmonary edema, etc. The pathogenesis is complex and is generally considered to be closely related to infection, atrial fibrillation, and heart rate arrhythmias. It has been found that once AMI occurs, it can lead to progressive left ventricular dilatation reconstruction, which is an important mechanism accompanying heart failure in patients with this disease and is an independent marker of death in AMI patients [7–10]. Left ventricular remodeling mainly includes the following aspects: (1) secondary dilatation of distant noninfarcted hypertrophic myocardium is seen; (2) expansion of the infarct zone occurs; (3) fibrosis of the myocardial interstitium occurs and the contractility is significantly reduced; (4) spherical changes in the left ventricular structure, i.e., a tendency to spherical shape from the original normal long oval shape [7–10]. Clinical treatment of AMI mostly focuses on controlling blood pressure, anti-infection, maintaining blood circulation, and controlling blood glucose to correct the patient's cerebral hypoxia and ischemia, which helps to control the degree of brain injury in order to reduce mortality [11]. After the onset of AMI patients, their neuroendocrine is in an activated state, and neurohumoral regulatory factors and matrix metalloproteinases all play an important role in left ventricular remodeling. Myocardial infarction occurs due to the synthesis and secretion of a large number of catecholamines, resulting in a continuous state of sympathetic overactivation, causing vasoconstriction and tachycardia, which can increase the myocardial ischemic burden and, to a certain extent, myocardial oxygen consumption, leading to further myocardial injury or necrosis and myocardial fibroblast proliferation, resulting in ventricular remodeling [12–15]. Thus, clinical treatment of AMI needs to focus on alleviating or reversing left ventricular remodeling.

RETRACTED

In this study, the treatment group was treated with enalapril combined with bisoprolol, and the results showed that 93.55% of the total effective rate in the treatment group was higher than 67.74% in the control group; the LVEF level at 3 months after treatment was higher in the treatment group than in the control group, and the LVED, LVES, and LVM levels were lower than those in the control group; the incidence of 12.90% adverse reactions in the treatment group was lower than that of 16.13% in the control group, but the difference was not statistically significant. It is suggested that the combination of enalapril and bisoprolol in the treatment of AMI can promote efficacy and improve the cardiac function of patients without increasing the adverse effects, which can guarantee the safety of treatment. The reason for this is that enalapril is a kind of ACEI, which can inhibit the release of angiotensin II to control the abnormal sympathetic nerve activity, and at the same time, it can promote vasodilation, which is conducive to increasing coronary artery perfusion in the infarct area and achieving the purpose of reducing the heart burden. In addition, enalapril administration strengthens ventricular systolic function and reduces the risk of myocardial ischemia-reperfusion [16]. Bisoprolol, as a highly selective *β*-blocker, has a higher cardioselectivity and longer effective duration of action after administration, which can produce inhibition of sympathetic nerve activity, induce a decrease in heart rate and prolong ventricular diastole for the purpose of improving myocardial blood supply, which can limit the infarct size and reduce arrhythmic conditions. In addition, bisoprolol modulates the pressure reflex mechanism mediated by the vagus nerve and blocks the myocardial toxic effects of early overactivated sympathetic nerves in patients with AMI to improve myocardial remodeling [17]. NT-proBNP is currently recognized as one of the semester markers of heart failure and can be secreted in large amounts once neurosecretory activation occurs, and neuroendocrine activation can directly lead to increased risk of heart failure [18–20]. Both CRP and IL-6 are proinflammatory response factors, which can reflect the degree of inflammatory response stimulation in AMI, and have a certain predictive effect on prognosis [21]. This study found that the levels of NT-proBNP, CRP, and IL-6 in the treatment group were lower than those in the control group 3 months after treatment, suggesting that enalapril combined with bisoprolol in the treatment of AMI can improve the inflammatory response. Analysis of the reasons, bisoprolol can reduce sympathetic nerve activity, promote the improvement of myocardial diastolic function, reduce myocardial oxygen consumption, and at the same time can regulate the level of myocardial *β*1 receptors, achieve the purpose of improving myocardial autonomic regulation, reduce myocardial damage, and then downregulation of NT-proBNP, CRP., and IL-6 expression [22, 23]. SOD is a kind of metalloprotease, a natural oxygen free radical scavenger, which can accurately predict the oxidative stress state of the body, and its level is proportional to the anti-peroxidation ability of cardiomyocytes. MDA is a membrane lipid peroxidation product, which can free proteins and amino acids, promote the cross-linking of the above products, damage the vascular basement membrane, increase its thickness, and aggravate the degree of oxidative stress in the body. This study found that the SOD level in the treatment group was higher than that in the control group 3 months after treatment, and the MDA level was lower than that in the control group. Analysis of the reasons shows that after administration of bisoprolol, it can activate the activity of SOD, reduce the MDA produced by tissue hypoxia, improve arterial blood flow, and promote vasodilation in ischemic sites to protect cardiomyocytes [24, 25]. Secondly, the drug absorption and utilization rate of enalapril is high, and it can be rapidly hydrolyzed into enalapril after entering the human body, which is beneficial to reduce the vascular resistance of the body, so as to promote vascular expansion, increase cardiac output, and improve oxidative stress. The purpose of the state can eliminate MDA and regulate vascular endothelial function. The authors analyzed that the combination of enalapril and bisoprolol in the treatment of AMI can improve the efficacy, but the safety of drug combination therapy and monotherapy is not clear, which may be due to the small number of samples selected in this study.

RETRACTED

Taken together, the application of enalapril in combination with bisoprolol for AMI promotes improved efficacy, facilitates improved cardiac function, and promotes the reduction of inflammatory response and oxidative stress.

## Figures and Tables

**Figure 1:** Treatment effectiveness.

**Figure 2:** Cardiac function.

**Figure 3:** Inflammation indicators.

**Table 1:** Oxidative stress index comparison in the two types of groups ($\bar{x}\pm s$).

Time	Group	SOD (IU/ml)	MDA (nmol/ml)
1d before treatment	Control group (*n* = 31)	65.58 ± 7.15	6.55 ± 0.88
	Treatment group (*n* = 31)	65.29 ± 7.54	6.57 ± 0.79
*t*		0.155	0.094
*P* value		0.877	0.925

3 months after treatment	Control group (*n* = 31)	89.54 ± 10.29	5.11 ± 0.42
	Treatment group (*n* = 31)	104.26 ± 9.78	4.01 ± 0.66
*T*		5.773	7.828
*P* value		0.001	0.001

**Table 2:** Adverse reactions situation comparison between two sets of groups (*n* (%)).

Group	Number of cases	Low blood pressure	Sinus bradycardia	Cough	Rash	Incidence
Control group	31	1 (3.23)	1 (3.22)	2 (6.45)	1 (3.23)	5 (16.13)
Treatment group	31	1 (3.22)	1 (3.23)	1 (3.22)	1 (3.23)	4 (12.90)
*X* ^2^						0.130
*P* value						0.718

## Data Availability

All the data generated or analysed during this study are included in this published article.
